This article has been retracted.

# Salidroside inhibits the proliferation and migration of gastric carcinoma cells and tumor growth *via* the activation of ERS-dependent autophagy and apoptosis

**DOI:** 10.1039/c9ra00044e

**Published:** 2019-08-15

**Authors:** Wei Yan, Kai Li, Amin Buhe, Tianxiong Li, Peirong Tian, Jun Hong

**Affiliations:** Department of General Surgery, Beijing Shijitan Hospital, Capital Medical University China wei_yan1@aliyun.com; Department of Surgery, Vanderbilt University Medical Center USA

## Abstract

The endoplasmic reticulum stress (ERS)-induced autophagy and apoptosis are favorable for the suppression of many cancer types. Salidroside (Salid) has been proven to be capable of inducing the apoptosis of many cancer cells. However, the underlying mechanisms and whether Salid can activate the autophagic system have still not been explained thoroughly. Herein, the inhibition effect of Salid on the growth and progress of gastric cancer and the underlying mechanisms were investigated. With the SGC-7901 cells acting as the cancer model cells, we ascertained that Salid exerted a superior antagonism effect on the growth and migration of gastric cancer cells in a dose-dependent manner. Additionally, Salid exhibited strong capacity to induce cell apoptosis by the down-regulation of proliferation-related genes (Ki67 and PCNA), increase in the pro-apoptotic protein C-caspase-3, and changing the levels of other related genes. A mechanism study revealed that the levels of the ERS-related genes, such as CHOP, C-caspase-12, GADD34, and BiP, in the SGC-7901 cells dramatically changed post-treatment by Salid, indicating the involvement of ERS in Salid-inducing cell apoptosis. In addition, the increased LC3^+^ autophagic vacuoles, enhanced conversion of LC3-I to LC3-II, and inhibition of the PI3K/Akt/mTOR pathway further confirmed the activation of autophagy induced by Salid. Importantly, the effect of Salid in regulating the levels of autophagy-related proteins or the signaling pathway could be markedly depressed by co-incubating with Wortmannin (Wort), an autophagy inhibitor. The final evaluation of the tumor therapy efficacy exhibited satisfactory cancer growth inhibition by Salid with negligible toxicity to normal tissues. In summary, the present work provides a comprehensive effective evaluation of Salid for treating gastric cancer. The detailed investigation of the underlying mechanisms may offer a rational reference for the future applications of Salid in clinic.

## Abstract 2

The endoplasmic reticulum stress (ERS)-induced autophagy and apoptosis are favorable for the suppression of many cancer types.

## Introduction

Gastric carcinoma (GC), one of the predominant causes of cancer-related deaths, is highly prevalent in humans all around the world and is generally characterized with a dismal prognosis.^1^ The main reason for gastric cancer being the fourth most frequent cancer and the fifth highest mortal malignant tumor is ascribed to its difficult diagnosis.^2^ The specific symptoms can rarely be efficiently detected by the existing techniques irrespective of whether it is the early stage or the later stage of gastric cancer.^3^ In this case, gastric cancer is often diagnosed at an advanced stage in the clinic, which always results in the failure of chemotherapy. Although laparoscopic-assisted surgery has widely demonstrated safety, feasibility, and favourable oncological results, the survival of gastric cancer patients post-operation is still unsatisfactory.^4–6^

Endoplasmic reticulum stress (ERS) is always induced during tumor development and progression and has become one of the most pivotal hallmarks of many malignancies.^7^ Although the ERS-induced unfolded protein response (UPR) program is a key prosurvival process, cell death induction results from sustained or prolonged stress.^8^ Importantly, ERS is the most important regulatory factor that activates autophagy and apoptosis.^8^ Considerable evidences have demonstrated that the ERS-dependent autophagy and apoptosis play key roles in the regulation of the programmed cell death of various tumor cells.^9,10^ Based on this, ER stress-induced autophagy and/or apoptosis have been widely investigated for the drug design and development of anticancer strategies.^11,12^

Salidroside (Salid), which is the main active ingredient of *Rhodiola rosea*, is commonly used for relieving high altitude sickness and replenishing vital energy.^13^ However, increasing number of studies have demonstrated that Salid can be an efficient anticancer drug due to its ability to inhibit the growth of bladder tumors through the activation of ERS.^14^ An investigation of the crosstalk between Salid and ERS manifested that Salid induced cancer cell apoptosis and restrained progress mainly by regulating the signaling pathways of AMPK/mTOR.^15^

Although numerous studies have demonstrated the capacity of Salid to suppress cell proliferation, promote apoptosis, and arrest the cell cycle of many tumor cells, such as bladder, breast, lung, and liver cancer cells,^16,17^ the complete understanding of the mechanism of the anti-gastric cancer effect of Salid remains elusive. In the present study, a comprehensive analysis of the effect of Salid on inhibiting gastric cancer was conducted by both cellular and animal assays. Moreover, the underlying mechanisms of Salid suppressing cancer cell proliferation and tumor growth were further evaluated by the corresponding experiments.

## Materials and methods

### Materials and cells

Salidroside and Wort were purchased from Meilun Biotechnology (Dalian, China). All primary and secondary antibodies were obtained from Abcam (Cambridge, MA, USA). The cell counting kit-8 (CCK-8) was bought from Dojindo Laboratories (Kumamoto, Japan). Plastic cell culture dishes, plates, and flasks were purchased from Corning Incorporation (Lowell, MA, USA). The 0.2% Triton X-100 was purchased from BD Bioscience (San Diego, CA, USA). Dulbecco's modified Eagle's medium (DMEM) was purchased from Gibco (Grand Island, NY, USA, #11765-054). Fetal bovine serum (FBS), penicillin/streptomycin, and M-PER Mammalian Protein Extraction Reagent were all obtained from Thermo Fisher Scientific (Waltham, MA, USA). All other chemicals were of analytical reagent grade and used without further purification.

The human gastric cancer cell line SGC-7901 was obtained from Shanghai Baili Biological Technology Co., Ltd. (Shanghai, China). Cells were incubated in complete DMEM containing 10% fetal bovine serum and supplemented with 100 U mL^−1^ penicillin/streptomycin.

### Animals and gastric cancer models

Sixty-four male nude mice (weighing 20–30 g each) were obtained from Shanghai Sino-British Sippr/BK Lab Animal Ltd. (Shanghai, China) and cultured under specific pathogen-free conditions. For the establishment of the gastric cancer-bearing mice models, the normal mice were anesthetized with 5% chloral hydrate, followed by intraperitoneal injection with 5 × 10^6^ SGC-7901 cells. Then, all of the mice, including the normal nude mice and tumor-bearing mice, were maintained under the standard conditions and supplied with sufficient water and food. All animal procedures were performed in accordance with the Guidelines for Care and Use of Laboratory Animals of Capital Medical University and the experiments were approved by the Animal Ethics Committee of Beijing Shijitan Hospital.

### Cell viability analysis

First, 100 μL of SGC-7901 cell suspension (5 × 10^3^ cells per mL) was seeded in 96-well chamber slides and allowed to grow for 24 h. Then, fresh DMEM culture media containing various concentrations of Salid were added into each well of the corresponding plates. Cells without the treatment of Salid were applied as the control group. After 48 h of incubation, 10 μL CCK-8 solution was added into each well, followed by incubation for 4 h. Finally, the absorbance values were examined using a universal microplate spectrophotometer (Beckman) with the detection wavelength set at 450 nm.

### Apoptosis

SGC-7901 cells were seeded in the six-well plates at a density of 5 × 10^4^ cells and allowed to grow overnight. Then, various concentrations of Salid were added into the plates and incubated with cells for 24 h. For the evaluation of the drug-induced cell apoptosis, a double-staining experiment was subsequently conducted according to the manufacturer's protocol. Finally, the cell samples were detected *via* flow cytometry (BD FACScan Flow cytometer, USA) to analyze the percentage of early apoptotic cells (PI negative cells) and late apoptotic cells (PI positive cells). Importantly, three independent experiments were performed for each group.

### Migration assay

For the transwell migration assay, the SGC-7901 cells with different treatments were seeded on the upper transwell chamber (Corning) containing DMEM with 0.5% FBS, and the lower chamber was filled with DMEM medium containing 10% FBS. After 24 h of incubation, the SGC-7901 cells on the lower surface of the insert were washed and fixed with 4% paraformaldehyde. After that, the SGC-7901 cells were stained with 0.1% crystal violet for 15 min. The number of migrated cells was observed using a light microscope (Zeiss).

### Cell proliferation assay

To investigate the effect of Salid on the proliferation rate of gastric cancer cells, the SGC-7901 cells were seeded in a 96-well plate at a density of 5 × 10^3^ cells per well. After 24 h of incubation, the old medium in each well was replaced with a fresh DMEM culture medium containing different concentrations of Salid (1 mM, 2.5 mM, and 5 mM). The cells without the treatment of Salid were used as the control. Then, the proliferation rate of the cells was determined at 48 h by the CCK-8 method as above.

### Effect of Wort on the anti-cancer efficacy of Salid

To evaluate the effect of the autophagy inhibitor Wort on the anti-cancer effect of Salid, SGC-7901 cells were seeded in each well of the six-well plates at a density of 5 × 103 cells per cm^2^. Then, the cells were divided into four groups: control (without treatment of Salid or Wort), Salid (treated by 5 mM Salid), Wort (treated by 10 mM Wort), and Salid + Wort (treated by 5 mM Salid and 10 mM Wort). Of great importance, Wort was added with Salidroside at the same time. After 48 h of co-incubation, the cells were collected and subjected to Western blot and immunofluorescence analyses. Moreover, the role of Wort in regulating the efficacy of Salid was further determined in the tumor-bearing mice by respectively co-injecting with Saline, Salid (50 mg kg^−1^), and Wort (100 mg kg^−1^) + Salid (50 mg kg^−1^).

### Immunofluorescence assay

After the SGC-7901 cells were respectively treated by Salid (5 mM), Wort (10 mM), and Salid (5 mM) + Wort (10 mM), the cells were treated with 0.2% Triton X-100 for 5 min at room temperature. Then, the cells were incubated with FITC-labeled primary rabbit anti-LC3 antibodies for 1 h. After the cell nuclei were stained by DAPI, the level of LC3 in each group was observed by a Zeiss LSM 510 confocal microscope and quantitatively analyzed through a flow cytometer (Cytomics™ FC 500, Beckman Coulter, Miami, FL, USA).

### Anti-tumor effect *in vivo*

Thirty-six tumor-bearing mice were randomly grouped (*n* = 12) and respectively treated by saline (Ctrl-SGC-7901), Salid (50 mg kg^−1^), and Wort (100 mg kg^−1^) + Salid (50 mg kg^−1^). The treatment was done repeatedly every two days in a week. Then, the mice were raised under the standard conditions with the survival time and tumor volumes of the mice in each group carefully observed. After a total 30 days of experiments, all the mice were sacrificed and the tumor tissues were photographed and collected for further investigations.

### Western blot analysis

To examine the protein expression levels of Ki67, caspase-3, PCNA, CHOP, cleaved caspase-12, GADD34, BiP, LC3, P62, Beclin1, PI3K, AKT, and mTOR on gastric cancer cells or tissues, Western blot analysis was conducted. For the cellular experiments, the SGC-7901 cells were seeded in a Petri dish and allowed to grow for 100% confluence. After the treatment of different concentrations of Salid, the SGC-7901 cells were washed three times with PBS (pH 7.4), followed by trypsinization for 1 min to obtain the cell pellets. Subsequently, the total protein samples were extracted by the M-PER Mammalian Protein Extraction Reagent and determined by a BCA protein assay kit (Thermo Scientific). After the cell lysis was separated with SDS-PAGE, they were transferred to the polyvinylidene difluoride (PVDF) membranes followed by incubation with Tris-buffered Tween 20 solution containing 5% BSA. Then, the primary antibodies that were diluted 1 : 500 were incubated with the membranes overnight under the temperature of 4 °C. To detect the levels of various proteins in the SGC-7901 cells, horseradish peroxidase-labeled secondary antibodies (1 : 5000 dilution) were allowed to interact with the samples for 2 h before evaluating the bands of interest under the Fluor Chem Imaging System (Alpha Innotech, USA).

For the examination of protein expressions in the tumor tissues, gastric cancer-bearing mice were euthanized and all of the tumor tissues were obtained. Thereafter, the obtained tissue samples were immediately subjected to isolation and homogenization in a buffer of 2% SDS lysis containing 100× protease inhibitor cocktail. After the total protein samples were collected by centrifugation, the expression levels of various proteins were investigated as above.

### Enzyme-linked immunosorbent assay (ELISA)

The concentrations of SOD and MDA in the SGC-7901 cells and gastric tumor tissues were determined using commercially available ELISA kits (Cusabio Biotech Co., Wuhan, China). The experiments were performed according to the manufacturer's instructions with the optical density examined at 450 nm through a microplate reader.

### Immunohistochemistry analysis of the expressions of Ki67, caspase-3, and PCNA

After the treatment of various concentrations of Salid, all of the tumor-bearing mice were sacrificed and the tumor tissues were collected, followed by immersing in 4% paraformaldehyde overnight. To prepare 6 μm sections, the fixed tissues were gradient dehydrated by sucrose solutions and then embedded in paraffin. The immunohistochemistry analysis was subsequently performed as follows: the prepared sections were dewaxed with xylene and dehydrated by different ratios of ethanol. To retrieve the antigen, a citrate salt solution was applied and incubated with the samples for 20 min. Subsequently, a solution of methanol/3% H_2_O_2_ (v/v, 1 : 1) was further used. After 15 min of incubation, the primary antibodies were introduced and interacted with the tissue samples for 1 h before the slides were blocked by a solution containing 5% BSA, 5% goat serum, and 0.1% NaN_3_. To visualize the protein expressions, the HRP-conjugated secondary antibodies were finally applied and the results were observed under an optical instrument after processing by a diaminobenzidine (DAB) substrate.

### TUNEL assay

After a course of treatment by Salid, the gastric cancer tissues were collected and subjected to sectioning at 5 μm. Then, the slides were fixed by acetone, followed by staining with terminal deoxynucleotidyl transferase and detection buffer under the guideline of manufacturers. Finally, the ability of Salid to induce tumor cell apoptosis *in vivo* was evaluated by determining the total number of TUNEL positive nuclei under an optical microscope and by comparing with the mice treated by saline.

### Histopathological evaluation

Mice were randomly divided into three groups as follows: healthy control group (treated by saline), SGC-7901 group (gastric cancer-bearing mice without any treatment), and Salid group (gastric cancer-bearing mice injected with Salid). For histopathological evaluation, organs including liver, lung, kidney, and colon of mice were obtained and fixed in 4% paraformaldehyde. Before the tissues were sectioned (thickness, 5 μm), the collected organs were embedded in paraffin overnight. Finally, H&E staining was performed according to the manufacturer's guideline and the results were analyzed under a light microscope (BX51; Olympus, Tokyo, Japan).

### Statistical analysis

The data are represented as the mean ± SD (standard deviation). Statistical analysis was performed by Student's *t*-test, while multiple group data were analyzed using one-way ANOVA. A value of *p* < 0.05 was considered as a statistically significant difference.

## Results

### Cytotoxicity of Salid against SGC-7901 cells

The cytotoxicity of Salid to gastric cancer cells was determined by the CCK-8 assay. As shown in Fig. 1B, Salid exhibits negligible toxicity to cells below the concentration of 0.5 mM. However, a significant decrease in cell viability could be achieved by elevating the concentration of Salid to 1 mM and the toxicity of the drug to the SGC-7901 cells displayed a dosage-dependent manner.

**Fig. 1:** Characterization of Salid and evaluation of its cytotoxicity to gastric cancer cells. (A) Chemical structure of Salid; its molecular weight is 300.3 Da. (B) Cytotoxicity of Salid to SGC-7901 cells post treatment of various concentrations of drugs (0, 0.05, 0.1, 0.25, 0.5, 1.0, 2.5, 5, 10, 25, 50, 100, and 250 mM). The results were determined by the CCK-8 method. *p < 0.05, compared with the control group.

To quantitatively analyze the Salid-induced cell apoptosis, a double-staining approach was applied. As clearly illustrated in Fig. 2A and B, the SGC-7901 cells treated by Salid show an obvious signal of early apoptosis compared with the control group. Importantly, the total amount of the apoptotic cells was proportional to the concentration of Salid, and the group incubated with 5 mM drug exhibited the highest apoptosis rate.

**Fig. 2:** *In vitro* evaluation of the therapy effect of Salid on gastric carcinoma cells. The SGC-7901 cells were seeded in plates or transwell and incubated with Salid at the concentrations of 1, 2.5, and 5 mM, respectively. The cells treated without drugs acted as the control group. (A) Drug-induced cell apoptosis was evaluated by the Annexin V-FITC/PI Apoptosis Kit using a flow cytometer. Data analysis was performed using Cell-Quest software. (B) Quantitative statistics of the apoptotic cells post treatment with various concentrations of Salid. (C) The invasion ability of Salid-treated SGC-7901 cells was examined by Transwell assays and compared with the control group. (D) Quantitative analysis of the ability of Salid to inhibit the SGC-7901 cell invasion. (E) Anti-proliferation capacity of Salid was evaluated by the CCK-8 method. (F) Corresponding gene expression post treatment with various concentrations of Salid, as determined by the Western blot assay. (G) Quantitative evaluation of the levels of Ki67, caspase-3, and PCNA in SGC-7901 cells post treatment. *p < 0.05, each treatment was compared with the control group.

### Salid significantly inhibited the migration of SGC-7901 cells

To evaluate the ability of Salid to inhibit cancer cell migration, a transwell assay was performed with Matrigel as a model of an extracellular matrix barrier. After the barrier enzymatically degraded, the tumor cells traversed the membrane and subsequently proliferated in a new location. As shown in Fig. 2C, the cells stained with crystal violet under the filters (invasive cells) are abundant in the image of the control group. However, the invasive cells visibly decreased with Salid treatment. Moreover, the inhibition effects of Salid were more obvious on increasing the concentration of the drug (Fig. 2D).

### Salid inhibited the growth of gastric cancer cells through the regulation of the proliferation-related proteins

CCK-8 experiments were adopted to evaluate the capacity of Salid to inhibit the growth of gastric cancer cells. As demonstrated in Fig. 2E, the SGC-7901 cells without any treatment exhibit the most rapid growth rate at any time point. In contrast, after the treatment with Salid, the cell growth rate significantly decreased and the proliferation inhibition ability could be enhanced by increasing the concentration of the drug. Subsequently, the underlying mechanisms were determined. As displayed in Fig. 2F and G, the levels of Ki67 and PCNA, which facilitate the proliferation of cancer cells, in SGC-7901 are dramatically down-regulated after the treatment with Salid. In contrast, the pro-apoptotic protein cleaved caspase-3 (C-caspase-3) exhibited obvious elevation in expression.

### Salid induced cell apoptosis through the activation of ERS-dependent apoptosis

To further clearly illustrate the underlying molecular mechanisms of Salid inducing apoptosis and the growth inhibition of gastric cancer cells, the ERS-dependent apoptosis-related genes were detected. As shown in Fig. 3A–C, the expressions of CHOP and C-caspase-12 are markedly enhanced after the treatment with Salid. Besides, the levels of CHOP and C-caspase-12 in the SGC-7901 cells were elevated on increasing the concentration of Salid. However, the detection of the pro-survival proteins exhibited that the treatment with Salid resulted in a severe lack of GADD34 and BiP in the SGC-7901 cells. Furthermore, the determination of superoxide dismutase (SOD) and malondialdehyde (MDA) displayed a distinct difference between the expressions of these two genes after receiving Salid therapy. As shown in Fig. 3D and E, the expression of SOD in gastric cancer cells is restrained after incubation with Salid, while the level of MDA increases, further indicating that Salid inhibited the growth of the SGC-7901 cells through the activation of ERS-dependent apoptosis.

**Fig. 3:** Evaluation of the levels of endoplasmic reticulum stress markers in SGC-7901 cells post treatment with Salid. (A) Western blot assay was applied to determine the expression of the RES-related pro-apoptosis factors (CHOP and C-caspase-12) and pro-survival molecules (GADD34 and BiP). (B and C) Quantitative study of the expression levels of CHOP, C-caspase-12, GADD34, and BiP post treatment with Salid. (D and E) The concentrations of SOD and MDA in SGC-7901 cells incubated with Salid were detected by qRT-PCR experiments. *p < 0.05, each treatment was compared with the control group.

### ERS-dependent autophagy was also activated after the gastric cancer cells were treated by Salid

To further investigate whether Salid could activate ERS-dependent autophagy, the expressions of autophagy regulatory genes, including LC3, P62, and Beclin1, in gastric cancer cells post-treatment were examined. As shown in Fig. 4A and B, high levels of LC3 II/LC3 I and Beclin1 can be observed in the cells treated by Salid. For the autophagy degradation substrate P62, the gene expression in the cells without any treatment was significantly higher than that in the cells incubated with Salid. These results together suggested that the autophagy in gastric cancer cells could be significantly evoked by the activation of ERS induced by Salid. Moreover, we also investigated the effect of Salid on the regulation of the PI3K/Akt/mTOR pathway, which plays a significant role in suppressing autophagy. As shown in Fig. 4C and D, obvious negative regulation of this pathway could be observed after the treatment by Salid, and the expressions of PI3K, Akt, and mTOR were remarkably depressed.

**Fig. 4:** Investigation of the underlying mechanisms of Salid-induced cell apoptosis. After the SGC-7901 cells were treated by various concentrations of Salid, the expressions of the autophagy pathway-related genes, including LC3, P62, Beclin1, PI3K, AKT, and mTOR, were determined. For further confirmation, the autophagy inhibitor Wort was adopted. (A and B) Expression of LC3, P62, and Beclin1 was determined by the Western blot assay. (C and D) The effect of Salid on the levels of PI3K, AKT, and mTOR in SGC-7901 cells was studied by Western blot analysis. (E and F) Expression levels of LC3, P62, and Beclin post treatment of the autophagy inhibitors. (G) Immunofluorescence analysis of the concentration of LC3 in cells using confocal microscopy. (H) Quantitative evaluation of the levels of LC3 by flow cytometry. *p < 0.05, each treatment was compared with the control group.

### Pre-treating cells with an autophagy inhibitor significantly impaired the effect of Salid

For further confirmation, the autophagy inhibitor Wort was applied to co-incubate with gastric cancer cells. Then, the expression levels of LC3, P62, and Beclin1 were determined by a Western blot assay. As shown in Fig. 4E and F, the levels of LC3 II and Beclin1 in the cells treated by 5 mM Salid are particularly higher than that in the other groups, indicating strong autophagic activity. In contrast, after the treatment with 10 mM Wort, the activation of autophagy was obviously depressed, and the levels of LC3 II and Beclin1 significantly decreased. Further verification was performed by an immunofluorescence assay. The cells in the group related to Salid treatment displayed the strongest green signal, while the fluorescence intensity of the cells treated by Wort was lower than that of the control cells (Fig. 4G and H).

### Anti-tumor effect of Salid *in vivo*

After receiving various treatments, the tumor volumes and survival curve of the mice were determined and compared with that of the control group (injection with saline). From Fig. 5A, we can clearly observe that the tumor volumes of the mice treated by Salid are significantly smaller than those of the control group. Besides, the tumor growth curve revealed that the SGC-7901 tumors in mice that were i.v. injected with Salid grew significantly slower than those treated by saline. For the determination of the medium survival time, it could be seen that the mice treated by Salid achieved a longer survival time than the mice injected with saline (Fig. 5C). The anti-tumor effect of Salid was further determined by a TUNEL assay. As exhibited in Fig. 5D and E, the tumor tissues treated by Salid exhibit a stronger apoptotic signal than the control ones. Taking these results together, we conclude that Salid has a significant effect on inhibiting gastric cancer growth and progress.

**Fig. 5:** Evaluation of the therapy effect of Salid on gastric carcinoma-bearing mice. The SGC-7901 tumor-bearing nude mice were randomly divided into three groups: one group received Salid (50 mg kg^−1^) therapy and the others were treated by saline and Wort plus Salid. (A) Photographs of excised tumor tissues post treatment with Salid and compared with the control. (B) Examination of tumor volume changes after receiving a course of Salid treatment and compared with the mice treated by Salid plus Wort and saline. (C) Kaplan–Meier survival curve of gastric carcinoma-bearing mice treated with Salid, Salid plus Wort, and saline, respectively. (D and E) Cell apoptosis induced by Salid was determined by a TUNEL experiment and the expressions of Ki67, caspase-3, and PCNA in tumor tissues post treatment were evaluated by immunohistochemical analysis. (F and G) The levels of LC3, P62, Beclin1, PI3K, AKT, and mTOR in tumor tissues post injection of Salid. (H and I) Concentrations of SOD and MDA in tumor tissues of Salid-treated mice evaluated by qRT-PCR experiments. *p < 0.05, each treatment was compared with the control group.

### Salid inhibited tumor growth through the activation of ERS-dependent apoptosis and autophagy

The results of immunohistochemistry analysis shown in Fig. 5D and E exhibit that the expressions of Ki67 and PCNA in the SGC-7901 tumor tissues dramatically decrease after treatment with Salid, while the level of Caspase-3 increases. To confirm whether ERS-dependent apoptosis was involved, the biomarkers of SOD and MDA were subsequently studied. As shown in Fig. 5H and I, the expression of SOD was significantly suppressed, while the level of MDA was up-regulated after being treated by Salid. These results together indicated that ERS-dependent apoptosis was involved in the process of Salid inhibiting gastric cancer growth and progress.

For the investigation of the ERS-dependent autophagy, the autophagic inhibitor Wort was added to each group. As shown in Fig. 5A–C, the anti-tumor effect of Salid can be significantly down-regulated by co-treatment with the autophagic inhibitor. Besides, the levels of LC3-II/I and Beclin1 in the Salid-treated mice were significantly lower than that in the group of Wort + Salid, while the expression of p62 exhibited opposite results (Fig. 5F). Furthermore, the suppression of the PI3K/Akt/mTOR pathway in tumor tissues after treatment by Salid could be relieved by the additional treatment of Wort. Taking the above results together, it could be concluded that Salid inhibited tumor growth through the activation of ERS-dependent apoptosis and autophagy.

### Histopathological analysis of organs post-treatment of Salid

To evaluate the toxicity of Salid to normal tissues, tumor-bearing mice were injected with the agents at a dosage of 50 mg kg^−1^ (BW), followed by H&E staining of the organs, including the liver, lung, kidney, and colon. For comparison, normal mice injected with saline and tumor-bearing mice that did not receive any treatment were also subjected to histopathological analysis. As shown in Fig. 6, compared to the normal group that was not treated by any anticancer agents, the SGC-7901 tumor-bearing mice displayed obvious gastric lesions, such as blurry gastric muscle layers, disruption of gastric glands, and exfoliation of the superficial gastric epithelium. Furthermore, there were apparent histopathological changes in the other organs of the tumor-bearing mice, including the liver, lung, and kidney. However, after the treatment with Salid, such lesions were significantly alleviated, indicating the excellent safety and efficacy of Salid.

**Fig. 6:** Safety evaluation of Salid treatment. Normal nude mice were randomly divided into three groups (*n* = 3): control group without any treatment, SGC-7901 cell-bearing mice, and normal mice receiving Salid treatment at a dosage of 50 mg kg^−1^. Then, all mice were sacrificed and the main organs including the liver, lung, kidney, and colon were collected, followed by histopathological analysis using the H&E staining assay.

## Discussion

Gastric cancer, developing from the lining of the stomach, remains the fourth most frequent cancer and one of the most lethal malignancies in the world over the past several decades.^18,19^ Importantly, the average prevalence and mortality rate of gastric cancer are still increasing every year and most patients are often diagnosed with advanced gastric cancer upon admission.^20^ The failure of the diagnosis of gastric cancer in the early stage is mainly due to the asymptomatic or nonspecific symptoms of this kind of cancer.^21,22^

Salid was isolated from the plant *Rhodiola rosea* and found to be a potent compound with several important biological properties such as antioxidant activity, anti-inflammatory activity, and cancer inhibition.^23,24^ Herein, we selected Salid as the anticancer model drug and evaluated its treatment efficacy on gastric cancer. We found that Salid decreased cell viability in a dosage-dependent manner and the gastric cancer cells incubated with Salid showed an obvious signal of early apoptosis compared with the control group. Subsequently, the effect of Salid on the proliferation of the SGC-7901 cells was determined by CCK-8 experiments. The results exhibited that the cell growth rate significantly decreased post-treatment of Salid, indicating the excellent antiproliferation ability of Salid.

As a high-molecular-weight non-histone protein, Ki67 is supposed to be a critical factor for controlling the cell proliferation by affecting the cell cycle.^25^ Increasing evidences demonstrated that the overexpression of Ki67 in several cancers is related to the tumor progress and cell invasion.^25,26^ The sequential activation of caspase-3, one of the key mediators of apoptosis, plays a central role in the execution phase of cell apoptosis.^27^ PCNA is associated with promoting the proliferation of many cancer cell types, including gastric tumor cells.^28^ Based on this, we hypothesized that the regulation of cell proliferation-related gene expressions was involved in the process of Salid-induced gastric cancer cell apoptosis. As demonstrated by a Western blot assay, after treatment by Salid, the expression of the pro-apoptosis gene caspase-3 significantly increased, while the levels of Ki67 and PCNA decreased to a large extent.

The C/EBP homologous protein (CHOP), also known as growth arrest and DNA damage 153 (GADD153), is an important transcription factor that regulates apoptosis in response to ER stress.^29^ The activation of caspase-12 leads to the initiation of the proapoptotic caspase cascade, which is involved in the activation of caspase-3 and -7.^30,31^ Moreover, the overexpression of such pro-death protease has been detected on the surface of the ER membrane and can be activated by ER stressors.^32^ The DNA damage-inducible protein GADD34/MyD116 is a gene that can suppress cell growth and plays a critical role in ER-mediated cell death.^33^ In addition, GRP78/BiP has a cytoprotective effect in oncogenesis, and the overexpression of BiP has been reported to be closely related to the drug resistance of cancer.^34^ SOD represents an important enzyme that has protective effects on cancer cells against apoptosis resulting from oxidative stress, while the MDA content is always used as the definitive marker of lipid peroxidation.^35^ Taking these factors in consideration, an examination of the levels of CHOP, cleaved caspase-12, GADD34, BiP, SOD, and MDA was used for the evaluation of Salid-induced ER stress in this work. As clearly illustrated in Fig. 3, gastric cancer cells that have been incubated with Salid display higher levels of CHOP and cleaved caspase-12 expressions compared with the untreated ones. In contrast, the expressions of the pro-survival genes GADD34 and BiP in the SGC-7901 cells were markedly suppressed. Additionally, the expression of SOD in gastric cancer cells significantly decreased after treatment with Salid, while the level of MDA showed an opposite result. These results together demonstrated that Salid inhibited cell growth and migration through the activation of ER stress.

Autophagy represents one of the crucial regulators of cell survival in response to different stress conditions and has a great potential in the field of cancer treatment. It is now widely accepted that ER stress is the most potent trigger for the autophagy of many tumor cell types.^34^ As illustrated above, the activation of ER stress in gastric cancer cells was caused by the treatment with Salid. In this case, a mechanism of ERS-dependent autophagy activation might have evolved in the process of Salid-induced gastric cancer inhibition. To verify this, the autophagic marker genes including LC3-II/I^36^ and Beclin1 (ref. 37) were determined by Western blot experiments. As demonstrated in Fig. 4, the levels of LC3-II/I and Beclin1 are obviously elevated by the incubation of the SGC-7901 cells with Salid and the expression signal is proportional to the drug concentrations. In contrast, the expression of P62, which was identified as an autophagy adaptor and pro-oncogenic regulator,^37^ dramatically decreased after the treatment, indicating high activity of autophagy induced by the therapy of Salid. Furthermore, the PI3K/AKT/mTOR pathway, which has a vitally important effect on many cancer cellular processes such as apoptosis, transcription, translation, cell cycle progression and regulating autophagy,^38–40^ was determined. As confirmed by the examination results of gene expressions, the activation of the PI3K/AKT/mTOR pathway in gastric cancer cells was remarkably restrained after incubation with Salid.

The autophagy inhibitors, such as the siRNA of Atg5 or Atg7, are always used to investigate the role of autophagy in regulating cell processes.^41^ In the present study, we selected Wortmannin (Wort), a famous autophagy inhibitor, to confirm the effect of Salid on the regulation of ERS-dependent autophagy in gastric cancer cells. The results showed that co-incubation with Wort led to significant decrease in the autophagic marker gene expressions in the cells treated by Salid, suggesting that an autophagy activation process was involved in the therapy of gastric cancer by Salid.

Finally, the established gastric cancer-bearing mice were used to investigate the antitumor efficacy of Salid *in vivo*. After receiving a course of Salid treatment, the SGC-7901 tumors grew significantly slower than that in the control group. The Kaplan–Meier survival curves further displayed that the mice injected with Salid had the longest survival time. More importantly, the histopathological analysis of the organs obtained from the Salid-treated normal mice suggested satisfactory safety for the application of Salid in oncology.

## Conflicts of interest

The authors declare no competing financial interests.

## Abbreviations

ERS: Endoplasmic reticulum stress
Salid: Salidroside
GC: Gastric carcinoma
SGC: Gastric cancer cell lines
PCNA: Proliferating cell nuclear antigen
C-caspase-3: Cleaved caspase-3
SOD: Superoxide dismutase
MDA: Malondialdehyde

## Supplementary Material
